# Exercise Rehabilitation Improves Heart Function and Quality of Life in Elderly Patients with Chronic Heart Failure

This article has been retracted.

**DOI:** 10.1155/2022/8547906

**Published:** 2022-01-12

**Authors:** Xingyun Peng, Liuquan Tang

**Affiliations:** ^1^School of Smart Healthcare Industry, Chongqing City Management College, Shapingba 401331, Chongqing, China; ^2^The Department of Basic Education, Chongqing City Vocational College, Yongchuan 402160, Chongqing, China

## Abstract

With the acceleration of the aging process, there are more and more elderly patients with chronic heart failure. Chronic heart failure has severely affected the heart function and quality of life of the elderly. This article aims to study the further improvement of the heart function and the quality of life of elderly patients with chronic heart failure through exercise rehabilitation. In this paper, experimental analysis and comparative analysis are adopted, the experimental group and the control group are designed, the adaptive heart rate and breathing rate algorithm is adopted, the heart failure symptom assessment scale and the quality of life assessment tool are selected, and the two groups of different rehabilitation forms are compared. Data collection, sorting, and analysis of the patient's conditions are utilized. Through the use of exercise rehabilitation, the heart failure process will be slower and the recovery of heart strength will be faster than the control group. Before the experiment, the probability of shortness of breath in the two groups of patients with chronic heart failure symptoms was as high as 84.08%, and the symptom clusters were more serious; after the experiment, the SV and EF values after exercise rehabilitation were higher than those of the control group (*p* < 0.05). The quality of life in the realm, emotional realm, and other realms has been significantly improved. For elderly patients with chronic heart failure, reasonable exercise rehabilitation training can provide them with effective preventive measures and protective measures, improve the patients' heart function and quality of life, and play an important and key role.

## 1. Introduction

Chronic heart failure (CHF) is the initial myocardial infarction caused by some myocardial damage and other reasons, which leads to complex clinical symptoms. Myocardial infarction, myocardial disease, and overload of blood circulation mechanics (severe, myocarditis, etc.) can cause changes in myocardial structure and function and ultimately lead to a decrease in ventricular pump or filling function. Chronic heart failure is a disease with high morbidity and mortality. It is also the advanced stage of various cardiovascular diseases, which greatly reduces the quality of life and well-being of patients. The mortality of chronic heart failure is positively correlated with the age of the patients. In our country, as the aging of the population accelerates the process, the prevention and treatment of heart failure is an important public health issue.

Exercise rehabilitation is an effective secondary prevention measure for CHF patients. In 2013, according to the guidelines of the American College of Cardiology Foundation, rehabilitation training was recorded as an important recommendation for HR patients. Many foreign studies have shown that while reducing treatment costs, restarting exercise can effectively reduce the prevalence and mortality of heart failure, thereby improving the exercise resistance and quality of life of HR patients. In recent years, HR sports rehabilitation has developed in our country, but many medical staff still lack understanding of it. HR patients and their families cannot effectively use sports training for self-management and support. This article will observe the sports rehabilitation of HR patients, provide a basis for the sports rehabilitation of HR patients, and promote the development of cardiac rehabilitation training in China.

Ba proposed a deep learning system for sports injury medical rehabilitation based on MRI image analysis. Warm-up activities refer to a variety of physical exercises purposefully carried out before sports, training, and competitions in order to maximize physical activity and prevent injury preparations. Therefore, how to use MRI images for numerical analysis of the above tasks is very necessary. Combined with the deep learning model, a new image enhancement recognition model is proposed to undertake medical tasks. However, the medical rehabilitation cycle for sports injuries is long, and there are too many uncontrollable factors, which cannot guarantee the medical rehabilitation effect [1]. Mao et al. stated that chronic heart failure (CHF) is a clinical syndrome caused by a variety of cardiovascular diseases (CVDs), which is increasingly becoming the main cause of global morbidity and mortality. They have previously proved that a 4-day forest bathing trip can provide adjuvant treatment effects for CHF patients. In order to further study the duration of the effects of CHF patients and the optimal frequency of forest bathing, we recruited subjects who experienced forest bathing again after 4 weeks and randomly divided them into two groups, namely, the urban control group (city) and the forest bathing group (forest). After the second 4-day forest bathing trip, they observed that the levels of brain natriuretic peptide, a biomarker of heart failure, continued to decrease, and the inflammation and oxidative stress were weakened. Therefore, this exploratory study proves the additional benefits of two forest baths for elderly CHF patients, which will further pave the way for the analysis of the impact of such interventions on cardiovascular disease. However, their experimental subjects are relatively narrow, and the experimental results are not very representative [2]. Yu et al. investigated the characteristics of clinical treatment drugs for elderly chronic heart failure (CHF) with various degrees of renal failure. Elderly CHF patients who received treatment from October (2010) to October (2015) were selected, and retrospective case collection was used. The revised equation of diet therapy for kidney disease (MDRD) was used to study the spiral filtration rate. Patients were divided into normal renal function group, mild renal function group, and moderate to severe renal function group. The statistical analysis of the three groups of characteristic drugs was compared. Compared with the results of the normal renal function group and the mildly decreased group, the difference between the normal renal function group and the mildly decreased group was significant (*p* < 0.05). The use of ACEI and beta blockers from moderate to severely reduced groups is very small. Diuretics and spironolactone were used (*p* < 0.05). Compared with the normal renal function group, the use rate of ACEIs is low, and the use rate of diuretics is low. However, their experimental method has limitations and there are many restrictive factors [3].

The innovations of this article are as follows: (1) the adaptive heart rate and respiration rate algorithm is used to observe the patient's heart function data at any time during the exercise rehabilitation process to strengthen the monitoring of the patient's health; (2) theoretical analysis and empirical analysis are comparable. Theoretically combine the advantages of sports rehabilitation with the data of the research experiments in this article, and demonstrate the effects of sports rehabilitation.

## 2. Research Methods for Exercise Rehabilitation to Improve Heart Function and Quality of Life in Elderly Patients with Chronic Heart Failure

### 2.1. Chronic Heart Failure in the Elderly

Chronic heart failure (CHF) is a clinical syndrome caused by various heart abnormalities and dysfunctions caused by abdominal filling. This is the final stage formed by various heart diseases such as hypertension, valvular heart disease, and pulmonary heart disease [4]. According to the latest data, the incidence of heart failure in developed countries is 1.5%∼2.0%, and the incidence of people over 70 years old is 10%. A random sampling of urban and rural residents aged 35–74 in my country shows that the morbidity rate of heart failure is 0.9%, and the older the age, the higher the prevalence rate [5, 6]. The 3-year survival rate is only 44%, and the 5-year survival rate is equivalent to malignant tumors. At present, there are about 4 to 5 million patients with heart failure in our country, which has brought a huge economic burden to the society [7, 8]. Therefore, the symptom management of elderly patients with chronic heart failure has attracted the attention of medical staff.

Almost all CHF patients exhibit 2–9 symptoms at the same time during their illness, such as dyspnea, fatigue, edema, and other characteristic symptoms of heart failure [9, 10]. Pain, drowsiness, sadness and tension, loss of appetite, and other symptoms are related to underlying diseases, and psychological related symptoms such as restlessness and depression. These symptoms do not appear alone in the onset of the disease, but a variety of symptoms will appear at the same time, indicating the “symptoms” of the “complex” phenomenon of interaction [11, 12].

Regarding the treatment of the symptoms of heart failure patients, before the 1970s, CHF patients were considered necessary to restrict physical activity accompanied by exercise recovery and pain. However, prolonged rest may cause skeletal muscle atrophy, venous thrombosis, pulmonary embolism, pressure ulcers, reduced exercise tolerance, worsening symptoms, etc. [13, 14]. By 1979, studies pointed out that exercise rehabilitation was safe for CHF patients, and it was possible to improve the exercise resistance of CHF patients. In order to restore the motor function of CHF patients, many studies have been conducted overseas, and its effectiveness and safety have been confirmed to various degrees in China [15, 16]. In 2005, the European Society of Cardiology recommended exercise as an important part of cardiac rehabilitation training to stabilize patients with heart failure, as an effective secondary preventive measure. In the American College of Cardiology 2013 (ACCF)/AHA Heart Failure Management Guidelines, IA lists exercise rehabilitation training for heart failure recommended by patients with chronic heart failure [17, 18].

### 2.2. Sports Rehabilitation

Cardiac rehabilitation exercise refers to the use of various forms of exercise to improve cardiovascular and physiological functions, prevent or delay the onset of diseases, achieve the purpose of rehabilitation, reduce the risk of vascular events, and enable patients to obtain better functional status [19, 20]. Research and analysis believe that exercise recovery can improve vascular endothelial function, increase the strength of skeletal muscles, lower blood pressure, strengthen sympathetic nerves, improve exercise resistance, and increase skeletal creatinase activity [21, 22]. Possible effects include improvement in left ventricular excitation rate (LVEF) and final volume of left ventricular dilation, increase in heart rate, decrease in plasma neurohormonal levels, and changes in histological characteristics of skeletal muscle.

At present, there is insufficient demand for clinical rehabilitation training in sports activities in my country. Sports rehabilitation training is not recognized and evaluated by almost all hospitals and medical staff. Only a few hospitals and regions have developed sports rehabilitation [23, 24]. CHF patients have not yet received standard sports rehabilitation training instructions. The continuity and coordination of sports rehabilitation are is not strong, and many hospitals have increased the burden on patients, medical care, and social economy [25]. This article aims to provide beneficial clinical rehabilitation exercises for more heart failure patients with complex causes, multiple diseases, and low exercise capacity for elderly CHF patients and to explore effective forms of CHF exercise recovery to improve physical health. Provide theoretical support for the training effect of sports rehabilitation.

### 2.3. Quality of Life

Quality of life (QOL) is also called living conditions, including economic conditions, religious beliefs, emotions, physiology, psychology and society. Quality of life is a complex and multidimensional concept. There is no unified definition at present. It is divided into two research fields: health and nonhealth. Generally, it includes three aspects: happiness, subjective health, and the meaning of life.

Health-Related Quality of Life (HRQOL) is a subjective feeling. Compared with quality of life, the scope only relates to the health field, which specifically reflects the difference between the patient's actual functional status of the body and its expected functional status perception. Wenger believes that HRQOL has a multidimensional structure, which refers to the patient's subjective perception of the impact of physiological symptoms, health perception, and functional status on daily life. Physiological symptoms refer to disease-related symptoms and their effects on functional status and health perception; health perception is closely related to mortality and is similar to life satisfaction and happiness; functional status integrates self-care activities, interpersonal fields, social support, sleep, mental function, coping, and emotions.

The factors affecting the quality of life of patients with chronic heart failure are divided into four aspects: demographic sociological factors, disease-related factors, psychosocial factors, and other factors. (1) Demographic sociological factors research shows that the demographic sociological characteristics of patients with chronic heart failure, such as age, gender, personality traits, and marital status, are important factors affecting the quality of life. (2) Research on disease-related factors shows that the disease-related characteristics of patients with chronic heart failure, such as heart rate, heart failure type, cardiac function classification, ejection fraction, blood B-type Brain Natriuretic Peptide (BNP), symptoms, and comorbidities are important factors affecting the quality of life. The independent predictors of quality of life are gender, age, body mass index, systolic blood pressure, cardiac function classification, symptom burden, functional status, and use of Angiotensin-Converting Enzyme Inhibitors (ACEI) drugs. The functional status of elderly patients with chronic heart failure is poor, but their quality of life is better than that of young patients with low ejection fraction. The degree of damage to the quality of life is not related to ejection fraction. The relationship between quality of life and ejection fraction reflects the complexity of the development of symptoms in the process of chronic heart failure, suggesting that the understanding of symptoms needs to go beyond traditional pathophysiological models. (3) Psychosocial factors research shows that the psychosocial factors of patients with chronic heart failure, such as psychological distress, mental status, self-efficacy, social support, coping style, are closely related to the quality of life. (4) Other factors: studies have found that the self-management, disease knowledge, functional status, rehabilitation exercise, and other conditions of patients with chronic heart failure are related to the patient's quality of life.

### 2.4. Adaptive Heart Rate and Breathing Rate Algorithm

#### 2.4.1. Bayesian Principle

Bayes' theorem refers to the theorem of conditional or critical probability of random events *A* and *B*. Its conditional probability is expressed by

(1) $$\begin{array}{c} P\left(AB\right)=P\left(A\right)P\left(B|A\right)=P\left(B\right)P\left(A|B\right). \end{array}$$

In the formula, *P*(*A|B*) refers to the probability of occurrence of *A* under the condition that *B* occurs, and *P*(*B|A*) is the probability of occurrence of *B* under the condition of occurrence of *A*. We can use the formula of conditional probability to derive the Bayesian formula as

(2) $$\begin{array}{c} P\left(B|A\right)=P\left(A|B\right)\cdot \frac{P\left(B\right)}{P\left(A\right)}. \end{array}$$

In other words, *P*(*B|A*) can be calculated by *P*(*A|B*), *P* (*A*), and *P* (*B*). Suppose *B* is a probability space {*B*1, *B*2,…*Bn*} composed of mutually independent events. Then, it can be expanded in the form of full probability:

(3) $$\begin{array}{c} P\left(A\right)=P\left(A|B_{1}\right)P\left(B_{1}\right)+P\left(A|B_{2}\right)P\left(B_{2}\right)+\cdots +P\left(A|B_{n}\right)P\left(B_{n}\right). \end{array}$$

Bayesian formula is represented as formula:

(4) $$\begin{array}{c} P\left(B_{i}|A\right)=\frac{P\left(A|B_{i}\right)P\left(B_{i}\right)}{P\left(A|B_{1}\right)P\left(B_{1}\right)+\cdots +P\left(A|B_{n}\right)P\left(B_{n}\right)}. \end{array}$$

*P*(*Bi|A*) is often called the posterior probability, and *P*(*A|Bn*)*P*(*Bn*) is the prior probability. *P*(*Bi*) is called the basic probability. In this algorithm, the three important estimators in the Bayesian probability fusion algorithm are adopted.

#### 2.4.2. Adaptive Heart Rate and Breathing Rate

The adaptive process is a process of continuously approaching the target. The path it follows is represented by a mathematical model, which constructs a mathematical model of the patient's heart rate and combines the physiological characteristics of heart rate and breathing to form a signal monitoring process for analysis. In this algorithm, we will use a short window to continuously slide on the signal for iterative calculations. During each sliding process, the length of the heartbeat and breathing interval in the sliding window will be estimated, so we need to set the heartbeat and breathing separately. The expected heart rate range in this algorithm is 40–160 beats/minute; that is, the expected heartbeat interval min = 60/160 s, max = 60/40 s; the expected range of breathing is 6–40 beats/minute, which is expected. The respiratory interval min = 60/40 s, max = 60/6 s. In order to accurately detect the heartbeat and respiration, ensure that the sliding window contains at least two complete heartbeats or respirations, and the length of the sliding judgment window is at least two maximum intervals. Use *j* to represent the *j*-th sliding window, *mj* to represent the center of the *j*-th sliding window, gs to represent the sampling rate, and *x* (*m*) to represent the signal after signal preprocessing and filtering without body movement; then, the *j*-th window is expressed as

(5) $$\begin{array}{c} Q_{j}\left[b\right]=x\left[m_{j}+b\right],b\in \left\{-\max,g_{s},\cdots ,\max\cdot g_{s}\right\}. \end{array}$$

In this algorithm, we will evaluate each possible interval length of each analysis window *Qj*[*b*] of the heartbeat signal and breathing signal through three estimators (*M* ∈ {*M*_min_, ⋯, *M*_max_}, *M*_min_=*Y*_min_ · *g*_*s*_, *M*_max_=*Y*_max_ · *g*_*s*_), and calculate the most likely *Yj*.

*(1) Three Estimators Improve Autocorrelation*. Autocorrelation is widely used in signal processing, and the similarity of signals can be detected through autocorrelation. In this algorithm, we use a mature and improved autocorrelation function to estimate the length of each possible interval of each analysis window *Qj*[*b*] of the heartbeat signal and breathing signal. The autocorrelation function formula is shown in

(6) $$\begin{array}{c} T\left[M\right]=\frac{1}{M}\sum_{b=0}^{M}Q\left[b\right]Q\left[b-M\right]. \end{array}$$

*(2) Improve the Average Amplitude Difference*. The traditional average amplitude difference takes the minimum value of *Q*[*b*] − *Q*[*b* − *M*] when the signals are similar. This parameter can be used to infer the similarity of the signal. In this algorithm, we unify the value of the estimator and obtain the maximum value when the signal has high similarity, so the traditional average amplitude difference is reversed, so that it is unified with the values of other estimators and is convenient for analysis. The specific improved average amplitude difference formula is shown in

(7) $$\begin{array}{c} T_{\text{MDF}}\left[M\right]={\left(\frac{1}{M}\sum_{b=0}^{M}\left|Q\left[b\right]-Q\left[b-M\right]\right|\right)}^{-1}. \end{array}$$

*(3) Maximum Amplitude Pair*. The maximum amplitude pair is the best representation of the amplitude information of the signal. In the successive periods before and after the signal, the amplitude sum of *N* corresponding to the peak of the signal and the peak is the largest, which is beneficial to the direct detection of the signal peak. Because this estimator relies on the peak amplitude information of the signal, it is susceptible to the influence of signal quality, but it can greatly improve the accuracy of signal estimation while combining the first two estimates. The calculation formula of the specific maximum amplitude pair is shown in the following formula:

(8) $$\begin{array}{c} T_{\text{MAP}}\left[M\right]=\underset{b\in \left\{0,\cdots ,M\right\}}{\max}\left(Q\left[b\right]+Q\left[b-M\right]\right). \end{array}$$

In this algorithm, we will calculate three estimator values *b* ∈ {−*Y*_max_ · *g*_*s*_, ⋯, *Y*_max_ · *g*_*s*_} in different interval threshold ranges *M* ∈ {*M*_min_, ⋯, *M*_max_} for each sliding window *Qj*[*b*]. Calculate the most likely local signal interval length by combining the values of three different estimators at different points.

#### 2.4.3. Estimator Fusion

The estimator through the above calculation method provides a possible value of the interval at which each *M* is correct. In this algorithm, we look at the output of the above three estimators (autocorrelation, average amplitude difference, and maximum amplitude pair) separately. It is formed into three Bayesian posterior probability density functions. These three probability density functions describe the probability of each estimator so that its output *N* is the true signal interval length. The *N* with the highest probability is the most common interval length:

(9) $$\begin{array}{c} M=\underset{M}{\max}p\left(M|T,T_{\text{MDF}},T_{\text{MAP}}\right). \end{array}$$

According to the Bayesian principle, the probability density function can be described as

(10) $$\begin{array}{c} P\left(M|T,T_{\text{MDF}},T_{\text{MAP}}\right)=\underset{p\left(T,T_{\text{MDF}},T_{\text{MAP}}\right)}{p\left(T,T_{\text{MDF}},T_{\text{MAP}}|M\right)p\left(M\right)}. \end{array}$$

Assuming that the similarity between estimators is only related to the true interval length of the signal and not related to the output of other estimators, formula (10) can be simplified according to the Bayes principle as

(11) $$\begin{array}{c} P\left(M|T,T_{\text{MDF}},T_{\text{MAP}}\right)\infty p\left(T,T_{\text{MDF}},T_{\text{MAP}}|M\right)p\left(M\right). \end{array}$$

Using Bayesian principle again, we can get

(12) $$\begin{array}{c} p\left(M|T,T_{\text{MDF}},T_{\text{MAP}}\right)\infty p\left(T|M\right)p\left(T_{\text{MDF}}|M\right)p\left(T_{\text{MAP}}|M\right)p\left(M\right). \end{array}$$

Ignore the fixed factors that have nothing to do with *M* and use Bayesian formula to get

(13) $$\begin{array}{c} p\left(M|T,T_{\text{MDF}},T_{\text{MAP}}\right)\infty p\left(M|T\right)p\left(M|T_{\text{MDF}}\right)p\left(M|T_{\text{MAP}}\right)p{\left(M\right)}^{-2}. \end{array}$$

We regard *P* (*M*) as a prior probability with uniform distribution; then, formula (13) is simplified to obtain

(14) $$\begin{array}{c} p\left(M|T,T_{\text{MDF}},T_{\text{MAP}}\right)\infty p\left(M|T\right)p\left(M|T_{\text{MDF}}\right)p\left(M|T_{\text{MAP}}\right). \end{array}$$

The three posterior probability density functions can be calculated by the following formula:

(15) $$\begin{array}{c} p\left(M|T\right)=\overset{T\left(M\right)-\min\left(T\right)}{\sum_{n=0}^{K}\left[T\left(m\right)-\min\left(T\right)\right]}. \end{array}$$

By fusing the three estimators, the maximum probability *N* obtained is the maximum data length of the most likely local interval, and then it can be converted to the signal local interval time length by the following formula (13)

(16) $$\begin{array}{c} Y=\frac{M}{g_{d}}. \end{array}$$

## 3. Exercise Rehabilitation to Improve the Heart Function and Quality of Life of Elderly Patients with Chronic Heart Failure

This article conducted a research experiment to improve the heart function and quality of life in elderly patients with chronic heart failure. The experimental group and the control group were selected for comparative experiments. The experimental group adopted exercise rehabilitation and the control group adopted traditional rehabilitation methods to compare the performance between the two groups. Changes in heart function and improvement in quality of life were noticed. This article selects heart failure symptom assessment scale and quality of life assessment tools to investigate from physical, emotional, and other fields. The experimental results show that exercise rehabilitation is beneficial to the recovery of heart function in elderly patients with chronic heart failure, and it can also improve the quality of life of patients and life happiness.

### 3.1. Experimental Research Objects

In this experiment, a total of 163 patients who were diagnosed and hospitalized in the Department of Cardiology, Geriatrics, and Cardiology Rehabilitation Department of Y Hospital from March (2019) to July (2019) were selected. It is divided into experimental group and control group. The experimental group takes the form of exercise rehabilitation, and the control group takes traditional rehabilitation. Through comparative experiments, the cardiac function and quality of life of the two groups of patients are studied.  Table 1 shows the inclusion and exclusion criteria of experimental research objects.

The included experimental subjects of heart failure patients must be unconscious and have basic communication skills. In addition, their participation in this trial has been approved by their family members. Those with liver and kidney failure, advanced malignant tumors, and other serious diseases should be excluded. It is mainly aimed at the physiological and psychological states of these patients under different intervention periods.

### 3.2. Research Methods

1. Patient general information questionnaire: This questionnaire is designed by the author to understand basic information such as age, course of disease, prevalence, gender, education level, and other basic information of patients. Among them, the symptoms of elderly patients were collected specifically during the data collection process.
2. Heart failure symptom assessment scale: This scale selects MSAS-HF, which includes the patient's physical, psychological, and heart failure symptoms, and has more than 30 subitems for testing to understand whether the patient has heart failure, degree of heart failure, frequency of occurrence, distress, etc.
3. Quality of life evaluation tools: The quality of life evaluation tools for patients with chronic heart failure are divided into nonspecific quality of life evaluation tools and specific quality of life evaluation tools.

### 3.3. Experimental Process

Both groups of patients received physical rehabilitation training on the basis of conventional drug treatment. The experimental group received sports rehabilitation, and the control group took traditional rehabilitation methods. The specific process is as follows:

  Experimental group: According to the different degrees of heart failure of patients, exercise training with different intensities is designed. The training mainly includes aerobic exercise; muscle strength training; flexibility training, including walking, jogging, Tai Chi, aerobic gymnastics; and reasonable control of exercise duration; all exercises are carried out under no physical load, and exercise frequency is average exercise every other day making appropriate adjustments based on your physical condition.
  Control group: Traditional rehabilitation training adopts conservative treatment methods. Exercise is not suitable, and it is best to maintain a happy mood.

The whole process of exercise is monitored by adaptive heart rate and breathing rate algorithm, and the stroke volume (SV) and left ventricular ejection fraction (EF) of all patients before and after exercise are measured. And the patient wear a monitoring bracelet to keep abreast of their cardiac function status and record the mood status, changes in the situation, appetite, and other related indicators every day.

### 3.4. Investigation Method

This experiment explained the situation of all patients, signed an informed consent form, and completed the questionnaire independently. Researchers completed and sorted out the questionnaire on the spot to ensure the validity and completeness of the questionnaire.

### 3.5. Statistical Analysis

The experimental data in this article are all used SPSS17.0 for data sorting and analysis. The measurement data are expressed in *x* ± *s*, and some are expressed in medians. All data are valid; this article also uses multifactor analysis to analyze the impact on the quality of life of patients and heart function research.

## 4. Exercise Rehabilitation Improves Heart Function and Quality of Life in Elderly Patients with Chronic Heart Failure

### 4.1. Comparison of General Data of the Two Groups of Patients

General data and clinical data surveys were conducted on the 163 study subjects that were finally included. The results of the survey are shown in Table 2. Among them, males accounted for 53.37% and females accounted for 46.63%; the average age was (68.78 ± 8.65) years; the vast majority of the subjects had a high school or technical secondary school degree or above (61.96%); 93.25% of the subjects had a spouse; family monthly income was 98.16% of the subjects with more than 1,000 yuan; about two-thirds of the subjects with NYHA classification are at level II (66.87%); the medical payment method for the vast majority of subjects is medical insurance (98.69%). The number of study subjects over 5 years accounted for 76.06%; 89.57% of the study subjects had more than 1 comorbidity; nearly half of the study subjects were equipped with stents (47.24%); and the difference in baseline data between the two groups was not statistically significant, indicating that the two groups of studies had comparable objects.

Figure 1 shows the change process of a patient's heart failure. The leftmost is the initial symptom. With a partial infarction, after a few hours to a few days, the infarct area becomes larger, and then after a long time without treatment, the heart undergoes a global renewal (plastic). The whole process demonstrates the deepening of the disease of patients with chronic heart failure, which seriously affects the health of patients.

### 4.2. Symptoms of Elderly Patients with Chronic Heart Failure

It can be seen from Table 3 that the top 10 symptoms in elderly patients with chronic heart failure in descending order are shortness of breath (84.08%), leg and arm edema (75.13%), dizziness (62.18%), cough (50.74) %), palpitations (50.35%), lack of energy (44.78%), sleep awake at night (41.73%), difficulty breathing when lying down (40.34%), dry mouth (37.82%), and lack of appetite (35.83%). The median score for the severity and distress of the above symptoms is 2 to 3 points.

It can be seen from Figure 2 that the symptom group of the experimental group after exercise rehabilitation has been significantly improved. Not only the mental state has improved, but the mood is also relaxed, and it will not be so easy to feel sleepy, nervous, and sad. Compared with the control, the effect of the group after ordinary rehabilitation is much better, and the severity of the overall symptom group has been reduced. Therefore, the form of rehabilitation through exercise is conducive to the patient's mental, psychological, and physical recovery and brings the patient a good exercise, to improve the patient's quality of life.

### 4.3. Exercise Rehabilitation Improves Heart Function Changes in Elderly Patients with Chronic Heart Failure

We measured the ventricular systolic function of patients, and the test results are shown in Table 4. It can be seen from the table that the SV and EF values of the two groups of patients before and after rehabilitation are statistically different, and the SV and EF values of the experimental group after exercise rehabilitation are higher than those of the control group (*p* < 0.05). The difference in the original data between the two groups was not large. After the intervention of the test group, the maximum value of SV increased from 39.3 to 45.41; the maximum value of EF increased from 44.26 to 51.01. Regardless of SV or EF, the data of the control group and the experimental group have increased to a certain extent before the intervention, but it is obvious that the data presented by the test group have greater fluctuations, indicating that the left ventricular systolic function is more. With coordination, the patient's heart rate tends to move more toward the normal range, indicating that the intervention has a significant therapeutic effect on heart rate failure.

The results of disease characteristics classification variables are shown in Figure 3. Among all chronic heart failure patients, 47.1% of patients have normal BMI, and 39.4% of patients with chronic heart failure are diagnosed for the first time. (54.0%) The heart function is the most in grade III, accounting for 57.7%, the patients with two causes are the most, accounting for 54.7%, the patients with one disease account for 40.5%, and the patients using 5-6 drugs account for 66.4%. The continuous variable data of disease characteristics showed that the average systolic blood pressure of the patients was (133.82 ± 21.42), the average diastolic blood pressure was (80.81 ± 13.68), and the average ejection fraction was (43.42 ± 9.07).

Factors affecting their quality of life mainly include changes in their physiological functions, decreased exercise endurance (due to insufficient cardiac output and insufficient oxygen), high psychological stress (anxiety, depression), cognitive impairment, individual psychological characteristics (cardiovascular patients are affected by functional recovery impact), and lack of social support (burden and pressure on family members). According to the Pearson correlation analysis between the heart function indexes (6MWT distance, LVEF, NT-proBNP) of patients with chronic heart failure and the Minnesota heart failure quality of life scores, the results in Figure 4 show that the 6MWT distance and LVEF of elderly patients with chronic heart failure are related to the quality of life. Obviously it has negative correlation (*r* = −0.494/−0.385, *p* < 0.01); NT-proBNP is significantly positively correlated with quality of life (*r* = 0.331, *p* < 0.01).

### 4.4. Exercise Rehabilitation Improves the Quality of Life of Elderly Patients with Chronic Heart Failure

In order to verify the influence of other factors on the survey results, this paper assigns a single factor and introduces a multifactor logistic regression model for analysis. The assignment results are shown in Table 5.

The step-by-step method is adopted, with 0.05 as the significance level of the introduced variable and 0.10 as the significance level of the excluded variable. This is based on the algorithm of the expected range of heartbeat and respiration. In the previous article, the multifactor analysis method was used to estimate and predict the amplitude of this fluctuation. Pearson correlation analysis can provide sufficient basis for it. The results in Figure 5 show that the number of hospitalizations due to heart failure, self-care ability, cardiac function classification, anxiety, dyspnea, and comorbidities in the past year are independent factors affecting the quality of life of patients with chronic heart failure. The quality of life has a greater impact.

Two-factor (group factor and time factor) repeated measures analysis of variance was used to compare the differences in the total quality of life scores between the two groups of patients. The experimental results are shown in Figure 6. Group factors include test group and control group, and time factors include 5 levels (baseline, 1 month of recovery, 3 months of recovery, 6 months of recovery, and 12 months of recovery). The results of repeated measures analysis of variance showed that there were differences in the total quality of life scores between different groups (*F* = 11.48, *p*=0.001); there were differences in the total quality of life scores between different time points (*F* = 117.78, *p* < 0.001) and rehabilitation There is an interaction between method and time (*F* = 34.68, *p* < 0.001).

It can be seen from Figure 7 that the total quality of life of patients with chronic heart failure is (42.59 ± 10.62), the score in the physical domain is (18.45 ± 4.59), the score in the emotional domain is (10.39 ± 3.20), and the score in other domains is (13.74 ± 4.08). According to the quality of life, each dimension is equally divided; from high to low, they are the physical domain, other domains, and the emotional domain.

It can be seen from Figure 8 that according to the results of a single factor analysis of the quality of life of patients with chronic heart failure, the differences in the quality of life of patients with chronic heart failure in groups of different per capita income, first-visit heart failure, heart failure type, heart function classification, and combined different diseases are statistically significant (*p* < 0.05). The results show that different per capita income, heart failure at first diagnosis, and the number of combined diseases enter the regression equation, which can explain 14.8% of the variation in quality of life.

In order to further reveal the relationship between symptom burden, self-efficacy, social support, and quality of life, the quality of life is used as a dependent variable, with different per capita income, heart failure at first diagnosis, number of combined diseases and symptom burden, self-efficacy, and social support. Carry out regression analysis for the independent variables and incorporate all the independent variables into the regression equation. The results are shown in Figure 9. It can be seen from the results that symptom burden, self-efficacy, and social support can explain 59.8% of the variation in quality of life.

## 5. Conclusion

This article mainly focuses on the research of exercise rehabilitation to improve the heart function and quality of life of elderly patients with chronic heart failure. Through literature data method, experimental analysis method, and comparative analysis method, it shows that exercise rehabilitation can effectively improve the elderly patients with chronic heart failure. Cardiac function, self-efficacy, social support, and other aspects have been very effective, which can effectively improve the quality of life of patients. The innovation of this paper is to use adaptive heart rate and respiration rate algorithm to detect the heart function of the patient. While protecting the health of the patient, observe the changes of the patient's heart rate and other indicators to keep abreast of the patient's heart function. And this article has strong pertinence in topic selection and design, and it is original and innovative. The limitation of this article is that the sampling range is narrow, the representativeness of the sample is not strong, and the exercise risk is not accurately grasped, which limits the experimental process of the research object. Future research can expand the scope and age of research, increase the sample base, and make reasonable arrangements from a more professional sports rehabilitation perspective to ensure and improve the health of patients.

## Figures and Tables

**Figure 1:** Heart changes in patients with chronic heart failure.

**Figure 2:** Comparative analysis of the symptom cluster severity scores of the experimental group and the control group.

**Figure 3:** Results of continuous variables in the disease-related data of the research subjects.

**Figure 4:** Correlation analysis of heart function and quality of life in elderly patients with chronic heart failure.

**Figure 5:** Logistic analysis of factors affecting the quality of life in elderly patients with chronic heart failure.

**Figure 6:** Comparison of the quality of life scores of the two groups of patients after different recovery time.

**Figure 7:** The quality of life scores of elderly patients with chronic heart failure in different fields.

**Figure 8:** Multifactor analysis of quality of life in elderly patients with chronic heart failure.

**Figure 9:** Regression analysis of symptom burden, self-efficacy, social support, and quality of life.

**Table 1:** Inclusion and exclusion criteria of experimental research objects.

Standard	Detailed items
Inclusion criteria	According to the Chinese Guidelines for the Diagnosis and Treatment of Heart Failure (2014), CHF was diagnosed as CHF by a physician at or above the level of attending a cardiovascular specialist hospital, and it is in the I–IV grade according to the New York Heart Association (NYHA) heart function classification
	Age ≥60 years old
	Unconscious obstacles, with basic communication skills

Exclusion criteria	Patients after surgery such as heart transplantation or heart valve replacement
	People with mental illness
	People with cognitive impairment
	Accompanied by severe diseases such as liver and kidney failure, advanced malignant tumors, etc.
	Those who cannot understand or accurately provide relevant information

**Table 2:** Comparison of general data and clinical data of the experimental group and the control group.

Project	Category	Test group	Control group	*t*	*p*
Gender	Male	43	44	0.005	0.942
	Female	39	38		

Age	—	68.29	70.12	−1.638	0.064

Education level	Junior high school and below	31	32	1.403	0.496
	High school or technical secondary school	29	34		
	College degree and above	23	15		

Marital status	Married	77	74	0.085	0.772
	No spouse	5	6		

Family monthly income	＜1000	2	2	2.771	0.251
	1000–4000	68	63		
	＞4000	12	19		

Classification	II level	56	54	0.374	0.543
	III level	25	28		

Medical payment method	Public medical	18	16	0.454	0.797
	Medical insurance	59	59		
	Other	5	7		

Course of disease	1–3 year	19	22	0.256	0.613
	3–5 year	64	61		

Number of comorbidities	0	9	8	0.744	0.689
	1–3	46	52		
	3–5	27	23		

Whether it is equipped with bracket	Yes	41	36	0.717	0.392
	No	40	46		

**Table 3:** Symptoms in elderly patients with heart failure.

Sort	Symptoms	The occurrence of symptoms		Severity of symptoms	Level of distress
		*n*	Incidence	Median	Median
1	Shortness of breath	168	84.08	3	3
2	Edema of legs or arms	152	75.13	2	2
3	Dizziness	125	62.18	2	2
4	Cough	103	50.74	2	2
5	Palpitations	101	50.35	2	3
6	Exhausted	91	44.78	3	3
7	Sleep and wake up at night	85	41.73	3	3
8	Difficulty breathing when lying down	82	40.34	2	3
9	Dry mouth	77	37.82	2	2
10	Lack of appetite	72	35.83	2	2
11	Sweating	61	29.86	2	2
12	Chest pain	49	23.88	3	3
13	Trouble sleeping	46	23.36	3	3
14	Bloating	46	23.35	2	2
15	Nausea	28	13.42	2	0
16	Numbness in hands and feet	23	10.95	2	1.5
17	Decline in physical fitness	22	10.44	2	1
18	Hard to concentrate	18	8.45	2	2
19	Vomiting	15	6.96	2	2
20	Anxiety	15	6.96	2	2
21	Itchy skin	14	6.45	2	2

**Table 4:** Comparison of changes in left ventricular systolic function before and after rehabilitation between the two groups.

Group	Number of cases	SV (ml)		EF (%)	
		Before intervention	After the intervention	Before intervention	After the intervention
Control group	58	37.25 ± 3.32	41.38 ± 1.54	40.15 ± 5.56	45.12 ± 3.58
Test group	65	37.15 ± 2.15	43.2 ± 2.21	39.78 ± 4.48	46.82 ± 4.19

**Table 5:** Variable setting and assignment.

Variable name	Assignment
Number of hospitalizations due to heart failure in the past year	0 = 0; 1∼3 = 1; 3∼5 = 2
Heart function classification	II = 0; III = 1; IV = 2
Medical payment method	Medical insurance = 0; self-pay = 1
Whether it is equipped with bracket	No = 0; Yes = 1
Anxiety/depression	0∼7 = 1; 8∼10 = 2; 11∼21 = 3
Difficulty breathing	Yes = 1; No = 0
Edema	Yes = 1; No = 0
Complications	0 = 0; 1∼3 = 1; 3∼5 = 2
Heart failure quality of life score	≤30 = 0; >30 = 1

## Data Availability

No data were used to support this study.
